The article "A Review on Characteristics of Experimental Research on Acupuncture Treatment for Alzheimer's Disease: Study Design" was published in 2022. Journal: Evid Based Complement Alternat Med.

# A Review on Characteristics of Experimental Research on Acupuncture Treatment for Alzheimer's Disease: Study Design

**DOI:** 10.1155/2022/8243704

**Published:** 2022-07-09

**Authors:** Chao Ke, Shengtao Shan, Chuang Fang, Yewan Xia, Wei Zhang

**Affiliations:** The First Affiliated Hospital of Hunan University of Chinese Medicine, Changsha 410007, China

## Abstract

**Background:**

This review aims to systematically summarize and analyze recent high-quality animal research results about the use of acupuncture in Alzheimer's disease (AD) patients. This information will be useful in providing a reference for future experimental research and an experimental basis for the clinical use of acupuncture in the treatment of AD.

**Methods:**

We utilized and referenced various electronic libraries from their inception to November 2021. Relevant information was reviewed and information such as the journal names, publication records, animal model selections and preparations, intervention measures, acupoint selections, detection methods, and detection indicators was extracted. Results. A total of 75 eligible studies were selected for additional review. Male SAMP8 mice, APP/PS1 double transgenic mice, Sprague–Dawley (SD) rats, and Wistar rats were the four commonly used animal strains in the experiments. The animals were categorized as transgenic and surgical mouse models. Experimental interventions included manual acupuncture (MA), Electro-acupuncture (EA), Moxibustion, and EA combined with Moxibustion. A retention time of 20 min was the optimal timing for experimental studies, with 14 sessions chosen as the most common treatment time. EA was the most prescribed acupuncture treatment type with continuous wave, 2 Hz frequency, and 1 mA electric current selected as frequently used parameters. A total of 78 acupoint prescriptions were analyzed involving 21 acupoints. The top 3 combinations of common acupoints were GV20 ⟶ EX-HN3, GV20 ⟶ BL23, and GV20 ⟶ GV26. A total of 39 articles had positive drug control groups, sham acupuncture, and/or nonacupoint control groups. Furthermore, 10 types of behavioral tests, 29 detection methods, 178 evaluation indicators, and 18 tissue samples were included in the analysis.

**Conclusions:**

By collating these high-quality research studies systematically and comprehensively, acupuncture was found to be a viable and effective treatment in AD animal models. In addition, when designing experiments, researchers could refer to the detailed data provided here to make better schemes and maybe conduct more investigations in unresearched areas.

## 1. Introduction

Alzheimer's disease (AD), the most common neurodegenerative disorder in the world, is characterized by memory loss, cognitive dysfunction, and personality changes, resulting in high morbidity and health-care costs [1]. It was estimated that 65.7 million people will have lived with dementia worldwide by 2030, and 115.4 million in 2050 [2]. Currently, the global estimates of health-care-related costs for dementia are expected to exceed $2.54 trillion by the year 2030 [3]. Early diagnosis and treatment of AD will improve survival rate and lower institutionalization, in return reduce resource utilization and health care cost [4]. AD is widely recognized as an important public health issue requiring action to reduce its prevalence and improve medical treatment for those affected. To date, there is no cure for AD, and the underlying pathogenesis of the disease remains largely unknown. Acetylcholinesterase inhibitors (including rivastigmine, galantamine, and donepezil) and N-methyl-D-aspartate receptor antagonists (memantine) are the primary medications used for the treatment of AD that is capable of decelerating disease progression and providing symptomatic relief, albeit with inevitable side effects [5].

As an important part of Chinese traditional medicine, acupuncture has been used for the treatment of AD for a long time. The treatment is safe for treating AD patients and can improve AD patients' cognitive function and ability to carry out their daily tasks [6]. Many researchers have conducted considerable research on the use of acupuncture therapy in AD, with a large number of research studies published. In this review, we will summarize high-quality animal experimental research results from recent years, provide further analysis on valuable animal experiment details regarding the treatment of AD with acupuncture, and a resource for future exploration and an experimental basis for the clinical use of acupuncture in AD.

## 2. Methods

### 2.1. Research Strategy

We searched English electronic libraries including PubMed, Embase, and Web of Science, from their inception to November 2021. Mesh terms, Keyword, and abstract CONTAINS “electroacupuncture” OR “acupuncture” OR “acupuncture therapy” OR “acupuncture points” OR “moxibustion” OR “meridians” AND Mesh terms, Keyword, and abstract CONTAINS “Alzheimer Disease” OR “AD”.

### 2.2. Inclusion and Exclusion Criteria

The inclusion criteria were as follows:

① Type: Animal experiments. ② Model: The subject was a simple AD animal model. ③ Intervention: One of the following acupuncture therapies had to be included: acupuncture, electroacupuncture, moxibustion, or a combination of these methods. ④ Data source: Science Citation Index (SCI).

The exclusion criteria were as follows:

① Secondary research articles including reviews, systematic reviews, meta-analyses, physician experiences or case reports, theoretical discussions, commentaries, clinical research, dissertations, and conference papers were excluded from our analysis. ② For duplicate papers, the most recently updated version was utilized. ③ Manuscripts in which acupuncture treatment was not used were excluded. ④ Manuscripts where the data were unclear or the statistical methods used were inappropriate were not included in our analysis.

### 2.3. Data Extraction

Two reviewers recorded available information from included studies independently. Reviewers recorded information including journal names, publication records, animal model selections and preparations, intervention measures, acupoint selections, detection methods, and detection indicators for further analysis. The relevant information recorded was reviewed and extracted from the abstracts and full texts of included studies. Discrepancies in the collected data were settled by discussion. In cases of an unsettled dispute, an expert, Professor Zhang, was invited for arbitration.

### 2.4. Data Analysis

SPSS 18.0 software was used to analyze acupoint prescriptions. The apriori algorithm model was used to analyze the association rules of acupoint compatibility, which was calculated simultaneously with support degree, confidence degree, and rule support degree calculations. A network diagram of acupoint association rules was drawn to analyze the core acupoint matching prescription. We also used Gephi 0.8.2 software, a partition algorithm model was used to perform complex network analysis and to intuitively visualize the core acupoints in the prescription of acupoints illustrated with the help of a core acupoint association network diagram. We used two different methods of data mining to reflect the association comprehensively and objectively. All other analyses were performed using Microsoft Excel 2003 software.

## 3. Results

### 3.1. Study Selection

A total of 1139 records were identified from three electronic libraries including Embase (*n* = 348), PubMed (*n* = 220), and Web of Science (*n* = 571). After the screening of each of the articles, 75 eligible studies were selected for further analyses (Figure 1).

### 3.2. Publication Characteristics of Included Studies

Figure 2 shows the number of relevant articles selected by publication year. We observed a gradual upward trend in articles about the search terms beginning in 2012, with a peak observed in 2020. Of the 75 papers selected for our review, 35 were published in English language journals. *Evidence-Based Complementary and Alternative Medicine* (*n* = 9), *Neural Regeneration Research* (*n* = 8), and *Acupuncture in Medicine* (*n* = 7) ranked among the top three journals selected studies were published in (Table 1). The top three journals were published in 14 different countries, most commonly in the United States (*n* = 29), England (*n* = 13), Switzerland (*n* = 8), and India (*n* = 8) (Figure 3).

### 3.3. Overview of the Experimental Features of Included Studies

#### 3.3.1. Selection of Animals and Model Preparations

Table 2 summarizes the characteristics of the selected animals of included studies. SAMP8 mice (*n* = 31), amyloid precursor protein/presenilin 1 (APP/PS1) double transgenic mice (*n* = 17), Sprague–Dawley (SD) rats (*n* = 14) and Wistar rats (*n* = 6) were the four most common strains used in the experiments. Regarding gender, 53 studies used male animals, six studies used female animals, the use of both sexes was reported in four studies, and 12 studies did not disclose the gender of the animals used. The age ranges of animals in the selected studies varied considerably, ranging from 2 months to 24 months. When using Wistar rats, the ages of the rats are normally 2-month-old or 4-5-month-old, while SD rats are 3-month-old. 7-month-old or 8-month-old mice were commonly used in SAMP8 mouse studies, while 6-month-old or 7-month-old mice were commonly used in APP/PS1 double transgenic mouse studies.

Table 3 shows the demographic characteristics of each of the animal models utilized. Animals were roughly divided into transgenic or surgical mouse models. The transgenic mouse model group included SAMP8 mice, APP/PS1 double transgenic mice, presenilin 1 and 2 conditional double knockout (PScDKO) mice, 5x-familia-AD (5xFAD) mice, or Apolipoprotein *E* (APOE)-deficient mice. The surgical mouse model group included mice that underwent bilateral intraventricular injection of amyloid *β*-peptide1-42 (A*β*1-42), bilateral hippocampal injection of A*β* (A*β*1-40, A*β*1-42, or A*β*25-35), intraperitoneal injection of D-galactose (D-gal), left hippocampus injections of A*β*1-40, right NBM injection of ibotenic acid (IBA), bilateral basal nuclei injections of IBA or intragastric administrations of AlCl3. Based on these studies, transgenic mice typically simulated a model of AD with severe pathology.

Model verification (the methods used to determine if a rat is in AD condition) will determine if the modeling is successful. Of the 75 papers analyzed, 13 articles documented model validation, including seven using gene identification, three using a Y maze, two using a Morris water maze test, and one using an open field test. No details regarding model validation were mentioned in the remaining articles.

#### 3.3.2. Intervention Methods and Selection of Acupoints

Experimental interventions in selected studies included manual acupuncture (MA), electroacupuncture (EA), moxibustion, and EA combined with moxibustion. Fifty studies used EA, 19 used MA, five used moxibustion, and one used EA combined with moxibustion. Treatment duration ranged from 2 to 16 weeks, with retention time lasting from 10 to 30 minutes, and the length of treatment ranging from 14 to 72 sessions. Thus, a retention time of 20 min, treatment duration of 15 days, and treatments administered once a day for 14 sessions were the most commonly used parameters (Table 4).

Table 5 summarizes the parameters settings used during EA treatment. The Hans electronic acupuncture apparatus (*n* = 22) and G6805 acupuncture apparatus (*n* = 11) were the two most commonly used brands used to administer EA. Regarding waveform, continuous wave (*n* = 15) was the most commonly used, followed by sparse wave (*n* = 9). In terms of frequency, 2 Hz (*n* = 26) was utilized the most in the selected studies and 1 mA (*n* = 25) of electric current was most commonly used.

Table 6 summarizes the acupoints and acupoint prescriptions in the 75 selected studies. Acupoint frequency was analyzed based on the acquired 78 acupoint prescriptions, which involved 21 acupoints used a total of 182 times. Among the 78 acupoint prescriptions, a total of 58 multiacupoint prescriptions were selected for treatment, and 20 single-acupoint prescriptions were selected for treatment. The most commonly used multiacupoint prescriptions were “Baihui (GV20) + Yingtang (EX-HN3)+ Shuigou (GV26)”, and “Baihui (GV20) + Shenshu (BL23).” The top five acupoints with the highest frequency of use were Baihui (GV20), Yingtang (EX-HN3), Shenshu (BL23), Zu Sanli (ST36) and Shuigou (GV26). The most frequently used meridian was the governor vessel (GV), which was used 91 times and involved five acupoints. The distribution of acupoints used in mice is shown below (Figure 4).

We also analyzed the association rule of the combinations of common acupoints for the treatment of AD. There were nine acupoint combinations with confidence levels ranging more than 70% with a support degree of more than 12%. Of these, GV20 ⟶ GV26 and EX-HN3 had association rules of 100%, indicating that when GV20 was selected, the probability of selecting GV26 or EX-HN3 was 100%. In addition, the highest support degree was GV20 ⟶ EX-HN3, which was 26.92% (Table 7). The core acupoint association network of acupuncture for AD is listed in Figure 5. The degree of support from strongest to weakest was acupoint GV20 combined with EX-HN3, GV20 with BL23, and GV20 with GV26. Furthermore, we can also see the same result that the top three support degrees were GV20 ⟶ EX-HN3, GV20 ⟶ BL23, and GV20 ⟶ GV26 in Figure 6. We used two different methods of data mining to determine the association comprehensively and objectively. The results obtained by these two algorithms generated identical rankings(Table 6, Figures 5 and 6).

#### 3.3.3. Group Settings, Detection Methods, and Indicators

Table 8 describes the treatment group settings of the 75 included papers. Of the 75 manuscripts, only 13 papers included positive drug control groups, including 11 using donepezil hydrochloride, one using selegiline, and one using memantine. A total of 26 manuscripts included sham acupuncture or nonacupoint control groups. Key information regarding sham electroacupuncture control, nonacupoint control, and sham moxibustion control included current (needles were inserted without current), needling (penetrating or nonpenetrating the skin), acupoint (nonacupoint/irrelevant acupoint) and moxa (the moxa sticks were not ignited). A total of 9 sham operation groups were infused with saline or a water/acetonitrile mixture. Lastly, 12 other groups were included in the manuscripts based on the purpose of the experiment. For example, DNA methyltransferase (DNMT) inhibitors are used to verify DNA methylation mechanisms, and c-Jun N-terminal kinase (JNK) inhibitors are used to inactivate the JNK signaling pathway to investigate the effect of EA on cognitive impairment and the role of the JNK signaling pathway in AD.

In Table 9, the commonly used behavioral tests assessed in 68 articles are summarized, with one to three different behavioral tests used in each study. Of the 10 types of behavioral tests, the Morris water maze test (*n* = 61) was the most commonly used, followed by the novel object recognition task (*n* = 6) there included, with interleukin-1β, Y maze test (*n* = 6), open field test (*n* = 3), step-down avoidance test (*n* = 2), step-through test (*n* = 1), passive avoidance test (*n* = 1), escape/avoidance training (*n* = 1), and fear conditioning (*n* = 1), tightrope test (*n* = 1). Different evaluation indicators were used based on the different tests, with escape latency, platform crossing times, and time spent in the target quadrant being the most commonly used parameters (Table 9).

Biochemical detection assays were performed in 66 articles using 29 different detection methods. Western blot, immunohistochemistry, immunofluorescence staining, quantitative real-time polymerase chain reaction (RT-PCR), and enzyme-linked immunosorbent assays (ELISA) were the most prevalent. A total of 178 biochemical evaluation indicators were included, with interleukin-1*β* (IL-1*β*), A*β*1-42, A*β* being the top three indicators assessed. Across all studies, 18 tissue sample types were analyzed, with the hippocampus, cortex, and serum being the three most common sample types collected. Advanced technical evaluation methods were also widely used, including videography and electrophysiology detections (Table 10).

## 4. Discussion

Herein, we systematically and comprehensively summarized the details of the animal experiments performed in 75 selected studies. Our results revealed that transgenic mice were the most commonly used animal model. Studies have shown that in the hippocampus of 6-month-old SAMP8 mice, A*β* deposition comprised of clustered granules that contained A*β* 42, A*β* 40, and other A*β* protein precursor fragments, with deposition increasing in number and extent with age [7]. It was also found that extensive amyloid plaque deposition occurs in the brain of APP/PS1 double transgenic mice at 6 to 7 months of age [8]. Xuying Li et al. [9] observed the neurobehavioral and pathological characteristics of APP/PS1 double transgenic mice aged 7–10 months to evaluate the stability of the model, Cognitive dysfunction was found in 7-month-old mice, and A*β* deposition in the hippocampus and cortex of 10-month-old mice. This could account for the selection of 7-month-old and 8-month-old SAMP8 mice or 6-month-old and 7-month-old APP/PS1 double transgenic mice for a majority of AD-related studies. In contrast, 5xFAD mice begin to develop visible amyloid deposits as early as two months of age, and may therefore provide a model that better biologically reflects the course of AD than phenotypes in the APP/PS1 mouse model [10]. PScDKO mice also displayed obvious AD-like phenotypes, especially robust inflammatory responses both in the brain and in the periphery, however, no distinct changes in A*β* deposition were observed. For these reasons, the PScDKO mouse model is often chosen to study the effects of inflammation on the pathological processes of neurodegenerative diseases [11]. ApoE−/−mice fed high-fat diets had accelerated AD-like pathologies such as cognitive deficits; increased A*β*, phospho-tau (p-tau), and mortalin levels; microglial activation; and decreased nissl body numbers [12]. Therefore, special attention should be paid to the type of model, age of animals, and pathological mechanism it mimics when selecting the appropriate animal model for AD research. In our study, we identified only 13 articles describing model validation. However, model validation should be utilized in all studies to ensure the rigor and quality of the experimental findings.

According to our results, the hippocampus was the most commonly analyzed tissue sample. However, Khan et al. [13] have found that the entorhinal cortex was the first region of the brain affected in AD using high-resolution functional magnetic resonance imaging (fMRI) variant analysis. There is a neural projection between the prefrontal cortex and the hippocampus [14]. Simic et al. [15] reported that a dorsal raphe nucleus was closely related to the early stages of AD. It has previously been demonstrated that the lateral and medial parietal association cortex and lateral temporal cortex were most relevant to cognitive decline in AD [16]. In the review of these studies, we found very few manuscripts selected these tissues. Therefore, further studies should focus their efforts on analyzing pathologically relevant tissues to better our understanding of AD pathogenesis.

Based on our evaluation of indicators in the articles selected for this study, the most common topics in AD papers focused on A*β* peptide protein deposition and metabolism, neuroinflammation, oxidative stress, apoptosis, synaptic plasticity, tau phosphorylation, neurotransmitters, and brain-derived neurotrophic factors, glucose metabolism, brain responses, and autophagy. Our results are consistent with previous reviews [17,18]. Future studies should explore other relevant topics to provide more supporting evidence for the underlying mechanisms associated with acupuncture treatment for AD.

Our results also revealed that advanced technical means have been widely used to evaluate and investigate the mechanisms of acupuncture for AD treatment in recent years, especially functional brain imaging techniques, like positron emission tomography (PET), dynamic contrast-enhanced MRI (DCE-MRI), arterial spin labeling-fMRI (ASL-fMRI), magnetic resonance spectroscopy (MRS) [19–21] and electrophysiology [22]. These types of imaging-based research will provide novel opportunities to explore the underlying mechanisms of acupuncture in AD in a dynamic, visual, and objective manner [23].

Acupuncture is based on the theory of meridians and acupoints, and can adjust the balance of yin and yang to prevent and treat diseases. It is a useful form of complementary and alternative medicine that may work through different mechanisms and can reduce the side effects of traditional therapies [24]. However, it is worth noting that the efficacy of acupuncture depends on intervention time, acupoint selection, and treatment parameters, which should be considered when evaluating its benefits. We have the following three thoughts.

First, when is the best time to intervene with acupuncture in AD? In a study by Li et al. [25],4-month-old and 12-month-old APP/PS1 mice were used to simulate the mild and the moderate stages of AD, EA was found to be more effective in mild AD mice than in moderate AD mice by suppressing microglial polarization to the M1 phenotype and promoting microglial M2 polarization, they also found changes specifically in the number of A*β*-positive plaques, but not in the area fraction in moderate AD mice. Does this mean that acupuncture may only be beneficial in treating mild AD? To date, there is only one study that investigated this, and we were unable to draw clear conclusions from it. Yu et al. [26] previously determined that preventive EA treatment could attenuate dendritic spine loss and rescue neuronal microtubule injury when treatment was administered at acupoints on the first day after the injection of D-gal. This could indicate that earlier intervention may lead to better clinical outcomes. However, further studies are warranted to investigate this more deeply.

Second, what is the most preferred acupuncture point or prescription? In our study, we identified only two comparative studies of acupoint prescriptions. One study utilized the combination of acupoints GV20 and ST36, which outperformed treatment with GV20 or ST36 individually in aging rats by alleviating microbiota-gut-brain axis impairments and improving spatial learning and memory [27]. Another study demonstrated that EA at Sanyinjiao (SP 6) and Guanyuan (CV 4) can improve learning and memory abilities and hormone levels in the hypothalamic-pituitary-ovarian (HPO) axis, with EA-Sanyinjiao (SP 6) outperforming EA-Guanyuan (CV 4) [28]. Unfortunately, there are no current studies to date comparing different acupoint prescriptions for the treatment of AD. GV20, EX-HN3, BL23, ST36, GV26 are the commonly used acupoints used to treat neuropsychiatric disorders in our review. From the results of data mining, we found the top three combinations of common acupoints were GV20 ⟶ EX-HN3, GV20 ⟶ BL23, and GV20 ⟶ GV26. These acupoints all demonstrated promising efficacies based on the study results. Which single point would be better? Which combinations would be better? It is important to search for ideal acupoints or acupoint prescriptions that can provide a sufficient experimental basis for clinical acupoint selection and prescription composition for the treatment of AD.

Third, what are the optimal parameters for AD treatment? The results of our study showed that EA was the most commonly used acupuncture intervention method. EA has been widely used to treat neurodegenerative diseases [29]. A recent study showed that PEA alleviated cognitive dysfunction in rats with D-gal-induced aging compared with PMA [30]. MEA is an innovative therapy combining music therapy and EA that can help overcome acupuncture intolerability. A comparative study demonstrated that MEA performed better than EA in decreasing amyloid-beta levels in AD [31,32]. Frequencies between 2 and 5 Hz (low) and 50–100 Hz (high) are within the currently accepted frequency range for EA. It was found that the effects of EA at 50 Hz were better than that at two Hz in enhancing hippocampal synaptic transmission and in potentially improving memory disorders in AD rats [33]. Another study also showed that 50 Hz (High) EA was more effective than 2 Hz (low) or 30 Hz (medium) EA in protecting synapse-ultrastructure impairment [34]. Yang et al. [35] found that giving two courses of EA treatment and three courses of EA treatment led to different outcomes, after two courses of EA, no significant effects were observed in the number of senile plaques (SPs) or the expression of *β*-site APP-cleaving enzyme 1 (BACE1) and insulin-degrading enzyme (IDE) in the cortex, but three courses of EA has a significant effect on these parameters. Therefore, further investigations should focus on extending treatment times to assess the relationship between treatment time and the efficacy of EA.

The effects of EA depend on frequency, current, waveform, and duration of pulses (retention time, course of treatment). However, no studies have been performed to date comparing waveform and current parameters. According to our study results, treatment duration ranged from two to 16 weeks, treatment retention time lasted from 10 to 30 minutes and a total course of treatment ranged from 14 to 72 sessions. While only one study reported research on a treatment course, we identified no studies assessing the effects of retention time, which will require further investigation to better define clinical outcomes.

## 5. Conclusion

To our knowledge, this is the first study to summarize the high-quality animal experimental research results in acupuncture studies performed in recent years. By collating this literature, it is obvious that acupuncture was effective in ameliorating cognitive dysfunction in AD animals, and the treatment has progressed considerably in recent years. Through valuable animal experimental details, our study might aid future investigators in designing optimal experimental protocols and studies. Lastly, the work presented here may be used to identify current gaps in knowledge and guide future research in studies investigating the use of acupuncture for AD.

## Figures and Tables

**Figure 1:** Flow diagram of the study selection.

**Figure 2:** Overview of included studies by year.

**Figure 3:** Overview and map of included studies by country of publication.

**Figure 4:** The locations of 21 selected acupoints for AD treatment in included studies.

**Figure 5:** Association network graph of acupoint combinations in the treatment of AD with acupuncture (apriori-based algorithm). The width of the line indicates the support degree.

**Figure 6:** Core acupoint association network of acupoint combinations in the treatment of AD with acupuncture (partition-based algorithm). The size of the circle represents the frequency, and the width of the line indicates the support degree. Node value: 19. Edge value: 35.

**Table 1:** Overview of included studies by journal.

Journals	Studies,*n* = 75, *n*
Evidence-based complementary and alternative medicine	9*∗*1
Neural regeneration research	8*∗*1
Acupuncture in medicine	7*∗*1
Neural plasticity	6*∗*1
Frontiers in neuroscience	4*∗*1
Frontiers in aging Neuroscience, Journal of traditional Chinese Medicine, Medical science monitor	3*∗*3
BMC complementary and alternative Medicine, Behavioral Neurology, Molecular Neurobiology, Neuroreport, Journal of alternative and complementary medicine	2*∗*5
Free radical biology & Medicine, Frontiers in Pharmacology, Genes & diseases, Integrative medicine Research, Iranian journal of basic medical Sciences, Journal of Alzheimer's Disease, Journal of biomedical and translational Research, Journal of traditional Chinese medical Sciences, Journal of integrative neuroscience, Anatomical Record, Autophagy, Metabolic brain Disease, Molecular medicine Reports, Biological Research, Brain Research, Cellular and molecular biology, Neuropsychiatric disease and Treatment, Current alzheimer Research, Neuroscience Letters, PloS One, World journal of stem Cells, Journal of neuroinflammation	1*∗*22

a*∗*b, a means the number of articles in a journal, b means the number of journals.

**Table 2:** Animal selections.

Strain	Number of studies (*n*)	Sex (*n*)	Age (*n*)
SAMP8 mice	31	Male (27), female (1), unknown (3)	8 months (9), 7 months (8), 7.5 months (6), 4 months (1), 6 months (1), 10 months (1), 2/6/8/12 different months (1),7/9/11 different months (1), unknown (3)
APP/PS1 double transgenic mice	17	Male (12), female (1), unknown (4)	7 months (6), 6 months (4), 3 months (1), 4 months (1), 5 months (1), 9 months (1), 12 months (1), 4/12 different months (1), unknown (1)
SD rat	14	Male (8), half of each sex(2), female (1), unknown (3)	3 months (3), 2 months (1), 6 months (1), 22–24 months (1), unknown (8)
Wistar rat	6	Male (3), half of each sex(2), unknown (1)	2 months (2), 4–5 months (2), 12 months (1), unknown (1)
5xFAD mice	4	Male (1), female (3)	6.5 months (3), 5.5 months (1)
OLETF rat	1	Male (1)	3 months (1)
PScDKO mice	1	Unknown (1)	4 months (1)
ApoE−/−mice	1	Male (1)	2 months (1)

**Table 3:** Animal models.

Type (*n*)	Modeling method (*n*)	Model validation (*n*)
Transgenic model (54)	Directly select SAMP8 mice as model (31)	Gene identification (7), open field test (1), unknown (46)
	Directly select APP/PS1 double transgenic mice as model (17)	
	Directly select 5XFAD mice expressing gene mutations (4)	
	PScDKO mice by crossing the forebrain-specific PS1 heterozygous knockout mice with conventional PS2 heterozygous knockout mice (1)	
	Directly select ApoE−/−mice with high-fat diet as model (1)	
Surgical model (21)	Intraperitoneal injections of D-gal for 6 weeks + Bilateral hippocampal injections of A*β*1-40 (4)	Y maze (3), morris water maze test (2), unknown (16)
	Bilateral lateral ventricles injections of A*β*1-42 (3)	
	Bilateral hippocampal injections of A*β*1-40 (3)	
	Intraperitoneal injections of D-gal for 8 weeks (3)	
	Bilateral hippocampal injections of A*β*1-42 (2)	
	Intraperitoneal injections of D-gal for 6 weeks + Right NBM injections of IBA (2)	
	Left hippocampus injections of A*β*1-40 (1)	
	Bilateral hippocampal injections of A*β*25-35 (1)	
	Intraperitoneal injections of D-gal for 6 weeks + Bilateral basal nuclei injections of ibotenic acid (1)	
	Intraperitoneal injections of D-gal for 90 days + Intragastric administrations of AlCl3 for 90 days (1)	

**Table 4:** Treatment methods.

Treatment method (*n*)	Retention time (*n*)	Number of treatment sessions (*n*)	Treatment duration (*n*)
EA (50), MA (19), Moxibustion (5), EA + Moxibustion (1)	20 min (29), 15 min (17), 30 min (13), 10 min (5), unknown (11)	14 (15), 24 (14), 15 (12), 20 (6), 48 (5), 28 (4), 18 (3), 6 (3), 30 (2), 40 (2), 56 (2), 12 (1), 21 (1), 26 (1), 72 (1), unknown (3)	15 days, once a day, day 8 rest (12), 15 days, once a day (9), 4 weeks, once a day, 6 days per week (8), 4 weeks, once a day, 5 days per week (6), 30 days, once a day, 8 days of every 10 days (5), 4 weeks, once a day (4), 8 weeks, once a day, 6 days per week (4), 2 weeks, 3 days per week (3), 3 weeks, once a day, 6 days per week (3), 4 weeks, every other day (3), 8 weeks, once a day (2), 30 days, every other day (2),8 weeks, once a day, 5 days per week (2), 12 weeks, once a day, 6 days per week (1), 6 weeks, once a day, 5 days per week (1), 3 weeks, once a day, 5 days per week (1), 16 weeks, once a day, 3 days per week (1), 2 weeks, once a day, 6 days per week (1), 6 weeks, every other day (1), 3 weeks, once a day (1), 26 days, once a day (1), 30 days, once a day (1), unknown (3)

**Table 5:** Parameter settings for EA administration.

Brand (*n*)	Model (*n*)	Waveform (*n*)	Frequency (*n*)	Electric current (*n*)
Hans electronic acupuncture apparatus (22)	HANS-LH202 (14), HANS-100A (5), HANS-200 (3)	Continuous (15) sparse (9), disperse (4), sparse and dense (3), dense (1), unknown (21)	1/15 Hz (1), 80–100 Hz (1), unknown (4)	1 mA (25), 0.6 mA (5), 0.1 mA (5), 1.5 mA (2), ≤2 mA (2), 2 mA (2), 20 mA (1), 1–2 mA (1), 1–3 mA (1), 0.3 mA (1), unknown (8)
G6805 acupuncture apparatus (11)	G6805- II (5), G6805-2A (1), unknown (5)						
Other (20)	Hwato (5), ZJ-12H music EA device (2), Master-8 stimulator (2), Korean brand (2), unknown (9)						

**Table 6:** Acupoints and acupoint prescriptions of included studies.

Acupoint prescription (*n*)	Acupoint (*n*)	Meridian (*n*)
Single point (20),	GV20 (46), EX-HN3 (21),	GV (91)
GV20 + EX-HN3 + GV26 (12),	GV26 (13), GV24 (6), GV14 (5)	CV (32)
GV20 + BL23 (10),	CV17 (9), CV12 (9), CV4 (8),	BL (19)
GV20 + EX-HN3 (6),	CV6 (5), CV8 (1)	SP (12)
CV17 + CV12 + CV6 + ST36 + SP10 (5),	BL23 (18), BL17 (1)	KI (6)
RN17 + CV12 + CV4 + ST36 + SP10 (4),	SP10 (10), SP6 (2)	ST (13)
GV24 + GB13 (4), BL23 + GV14 (4),	KI3 (4), KI1 (2)	GB (4)
EX-HN3 + LI20 (3), GV20 + KI1 (2),	ST36 (13)	LI (3)
GV20 + GV24 (2), GV20 + GV26 (1),	GB13 (4)	PC (1)
GV20 + ST36 (1), GV20 + BL23 + KI3 (1),	LI20 (3)	HT (1)
GV20 + GV14 + BL23 (1),	PC6 (1)	
GV20 + BL23 + SP10 + BL17 (1),	HT7 (1)	
GV20 + BL23 + PC6 + ST36 + SP6 (1)		

**Table 7:** Analysis of the association rule of the combinations of common acupoints in treatment of AD with acupuncture.

Number	Acupoints	Cases	Support (%)	Confidence (%)	Rule support (%)	Lift
1	GV20 ⟶ EX-HN3	21	26.92	85.71	23.08	1.45
2	GV20 ⟶ BL23	18	23.08	77.78	17.95	1.32
3	GV20 ⟶ GV26	13	16.67	100.00	16.67	1.70
4	EX-HN3 ⟶ GV26	13	16.67	92.31	15.38	3.43
5	EX-HN3 ⟶ GV26 and GV20	13	16.67	92.31	15.38	3.43
6	GV20 ⟶ GV26 and EX-HN3	12	15.38	100.00	15.38	1.70
7	CV17 ⟶ SP10	10	12.82	90.00	11.54	7.80
8	CV12 ⟶ SP10	10	12.82	90.00	11.54	7.80
9	ST36 ⟶ SP10	10	12.82	90.00	11.54	5.40

By setting the minimum support >12% and the minimum confidence >70%, a total of nine sets of associated records were obtained.

**Table 8:** Experimental groups.

Treatment method (*n*)	Positive control groups (*n*)	Sham acupuncture groups or nonacupoint groups (*n*)	Sham-operated control groups (*n*)	Miscellaneous groups (*n*)
EA (50)	donepezil hydrochloride (7), memantine (1), selegiline (1)	Sham-EA (5), nonacupoint (6)	Equal volume of saline (7), equal volume of water/acetonitrile mixture (1)	Olfactory stimulation (2), Autophagy inhibitor (1), JNK pathway blocker (1), olfactory nerve cut group (1), DNMT inhibitor (1), NLPR3 inflammasome selective inhibitor (1), autophagy-lysosome pathway group (1)
MA (19)	donepezil hydrochloride (4)	Nonacupoint (13)	—	The neural stem cell (NSC) group (3), PDK1/nPKC/Rac1 inhibitor group (1)
Moxibustion (5)	—	sham moxibustion (2)	—	—
Moxibustion + EA(1)	—	—	Equal volume of saline (1)	—

**Table 9:** Behavioral tests.

Tests (*n*)	Evaluation indicators (*n*)
Morris water maze test (61)	Hidden platform trial: Escape latency (59), swimming distance (8), swimming speed (6).
	Probe trial test: platform crossing times (37), time spent in the target quadrant (26), ratio of swimming time in the target quadrant and total swimming time (13), ratio of swimming distance in the target quadrant and total swimming distance (5), swimming speed (5). Swimming distance in the target quadrant (4), latency to first target-site crossover (3), ratio of swimming time in every quadrant and total swimming time (3), number of entries to the target quadrant (1), time spent in the opposite quadrant (1).
	Reversal trial: Escape latency (4).
	Visible platform trial test: escape latency (3), swimming speed (1).
Novel object recognition task (6)	Percentage of new object exploration time/total exploration time (6), percentage of new object exploration numbers/total exploration numbers (2), percentage of old object exploration time/total exploration time (2), total exploration time (2).
Y maze (6)	Total reaction time (2), total entry frequencies in three arms (2), spontaneous alternations (2), duration in novel arm (1), frequency in novel arm (1), reaction time of getting learning skills (1)
Open field test (3)	Duration spent in the central zone (2), the frequency of crossing the central zone (1), distance in the central region (1), number of mice standing upright (1), activity distance (1).
Step-down avoidance test (2)	Latency period (2), number of errors (2).
Step-through test (1)	Mean number of errors of each group in the learning session (1), mean learning latency of each group in the learning session (1), mean number of errors of each group in the test session (1), mean test latency of each group in the test session (1).
Passive avoidance test (1)	Mean number of errors of each group in the learning session (1), mean learning latency of each group in the learning session (1), mean number of errors of each group in the test session (1), mean test latency of each group in the test session (1).
Escape/Avoidance training (1)	The number of escape responses (1), the response latency in escaping UCS shock (1).
Tightrope test (1)	Success rate (1).
Fear conditioning (1)	Percentage of animals frozen in the contextual test (1), percentage of animals frozen in cued test (1).

**Table 10:** Biochemical detection analyses.

	Tissue samples (*n*)	Tests (*n*)	Evaluation indicators (*n*)
Biochemical	Hippocampus (55), Cortex (8), serum (7), The frontal lobe cortex (6), prefrontal cortex (3), Cerebral cortex (2), Urine (2), Intestinal tissue (1), Dorsal raphe nucleus (1), Hypothalamus (1), Pituitary gland (1), Ovaries (1), Entorhinal cortex (1), cerebrospinal interstitial fluid (1), The parietal association cortex (1), stool (1), Cerebrospinal fluid (1), plasma (1)	Western blot (48), Immunohistochemistry (23), Immunofluorescence staining (19), RT-PCR (18), ELISA (14), Hematoxylin-eosin staining (10), Transmission electron microscopy (7), Nissl staining (6), TUNEL staining (4), Flow cytometry analysis (4), Immunoprecipitation (3), spectrophotometry (3), golgi staining (2), UPLC-MS (2), bisulfite sequencing (1), 16S rDNA amplicon sequencing (1), glucose oxidase method (1), GC-MS (1), Double-label immunofluorescence assays (1), BrdU staining (1), ROS staining (1), thioflavin staining (1), Colorimetric method (1), Optical fractionator method (1), Thiobarbituric acid method (1), Dithiodinitrobenzoic acid method (1), Xanthine oxidase method (1), Liquid chromatography-tandem mass spectrometry (1)	IL-1*β* (11), A*β*1-42 (11), A*β* (10), GFAP (10), BACE1 (8), Iba-1 (8), A*β*1-40 (7), p-Tau (7), GSK-3*β* (7), TNF-*α* (6), APP (6), IL-6(5), BDNF (4), ASC (4), p-GSK-3*β* (4), Caspasase-1 (4), AKT (4), PSD95 (4), synaptophysin (4), IL-10(3), tau (3), iNOS (3), p-AKT (3), AMPK (3), LC3B (3), NLRP1 (3), SOD (3), NLRP3 (2), p-AMPK (2), NeuN (2), IL-17(2), IL-18(2), BAX (2), IDE (2), MDA (2), Bcl-2 (2), TLR4(2), gut microbial (2), Arg1(2), SYN (2), LC3A (2), p-p38MAPK (2), Synapsin-1 (2), ATP (2), SIRT1 (2), APOE (2), PGC-1*α* (2), CD11 B (2), COX2(2), HO-1(2), transferrin (2), BAX (2), BrdU (2), other^a^ (125)
Other	—	Micro-PET (14), electrophysiology (3), Dynamic contrast enhancing (DCE)-MRI (1), arterial spin- labeling–functional MRI (ASL-fMRI) (1), MRI (1), MRS (1)	18F-FDG (14), fEPSP slope (2), signal intensity of ROIs (2), CBF (1), NAA/CrF (1), glu/CrF (1), MI/CrF (1), time-dependent anatomical routes of paravascular influx in the glymphatic system (1), I/O curve (1), LTP (1), Potentiation (1), PS amplitude of baseline (1)

Other^a^ includes 125 indicators, each appearing only once.

## Data Availability

The data used to support the findings of this study are available from the corresponding author upon request.

## References

[1] Alzheimer’s Association (2016). 2016 Alzheimer’s disease facts and figures. *Alzheimers Dement*.

[2] Prince M., Bryce R., Albanese E., Wimo A., Ribeiro W., Ferri C. P. (2013). The global prevalence of dementia: a systematic review and metaanalysis. *Alzheimer’s and Dementia*.

[3] Jia J., Wei C., Chen S. (2018). The cost of Alzheimer’s disease in China and re-estimation of costs worldwide. *Alzheimers Dement*.

[4] Black C. M., Fillit H., Xie L. (2018). Economic burden, mortality, and institutionalization in patients newly diagnosed with alzheimer’s disease. *Journal of Alzheimer’s Disease: JAD*.

[5] Kumar A., Singh A. (2015). A review on Alzheimer’s disease pathophysiology and its management: an update. *Pharmacological Reports*.

[6] Zhou J., Peng W., Xu M., Li W., Liu Z. (2015). The effectiveness and safety of acupuncture for patients with alzheimer disease. *Medicine (Baltimore)*.

[7] del Valle J., Duran-Vilaregut J., Manich G. (2010). Early amyloid accumulation in the hippocampus of SAMP8 mice. *Journal of Alzheimer’’ Disease*.

[8] Pistell P. J., Zhu M., Ingram D. K. (2008). Acquisition of conditioned taste aversion is impaired in the amyloid precursor protein/presenilin 1 mouse model of Alzheimer’s disease. *Neuroscience*.

[9] Li X., Guo F., Zhang Q. (2014). Electroacupuncture decreases cognitive impairment and promotes neurogenesis in the APP/PS1 transgenic mice. *BMC Complementary and Alternative Medicine*.

[10] Tohda C., Urano T., Umezaki M., Nemere I., Kuboyama T. (2012). Diosgenin is an exogenous activator of 1,25D3-MARRS/Pdia3/ERp57 and improves Alzheimer’s disease pathologies in 5XFAD mice. *Scientific Reports*.

[11] Jiang X., Zhang D., Shi J., Chen Y., Zhang P., Mei B. (2009). Increased inflammatory response both in brain and in periphery in presenilin 1 and presenilin 2 conditional double knock-out mice. *Journal of Alzheimer’s Disease*.

[12] Liu J., Zhao B., Cui Y. (2015). Effects of shenque moxibustion on behavioral changes and brain oxidative state in apolipoprotein e-deficient mice. *Evidence-based Complementary and Alternative Medicine: eCAM*.

[13] Khan U. A., Liu L., Provenzano F. A. (2014). Molecular drivers and cortical spread of lateral entorhinal cortex dysfunction in preclinical Alzheimer’s disease. *Nature Neuroscience*.

[14] Izaki Y., Takita M., Akema T. (2008). Specific role of the posterior dorsal hippocampus-prefrontal cortex in short-term working memory. *European Journal of Neuroscience*.

[15] Simic G., Stanic G., Mladinov M., Jovanov-Milosevic N., Kostovic I., Hof P. R. (2009). Does Alzheimer’s disease begin in the brainstem?. *Neuropathology and Applied Neurobiology*.

[16] Ossenkoppele R., Smith R., Ohlsson T. (2019). Associations between tau, A*β*, and cortical thickness with cognition in Alzheimer disease. *Neurology*.

[17] Song Y. Y., Xu W. T., Zhang X. C., Ni G. X. (2020). Mechanisms of electroacupuncture on alzheimer’s disease: a review of animal studies. *Chinese Journal of Integrative Medicine*.

[18] Yu C. C., Du Y. J., Wang S. Q. (2020). Experimental evidence of the benefits of acupuncture for alzheimer’s disease: an updated review. *Frontiers in Neuroscience*.

[19] Ding N., Jiang J., Xu A., Tang Y., Li Z. (2019). Manual acupuncture regulates behavior and cerebral blood flow in the SAMP8 mouse model of alzheimer’ disease. *Frontiers in Neuroscience*.

[20] Lin R., Li L., Zhang Y. (2018). Electroacupuncture ameliorate learning and memory by improving N-acetylaspartate and glutamate metabolism in APP/PS1 mice. *Biological Research*.

[21] Sun R. Q., Wang Z. D., Zhao J. (2021). Improvement of electroacupuncture on APP/PS1 transgenic mice in behavioral probably due to reducing deposition of A*β* in hippocampus. *The Anatomical Record*.

[22] Li K., Shi G., Zhao Y. (2021). Electroacupuncture ameliorates neuroinflammation-mediated cognitive deficits through inhibition of NLRP3 in presenilin1/2 conditional double knockout mice. *Neural Plasticity*.

[23] Yu C. C., Ma C. Y., Wang H. (2019). Effects of acupuncture on alzheimer’s disease: evidence from neuroimaging studies. *Chinese Journal of Integrative Medicine*.

[24] Park S., Lee J. H., Yang E. J. (2017). Effects of acupuncture on alzheimer’s disease in animal-based research. *Evidence-Based Complementary and Alternative Medicine*.

[25] Li L., Li L., Zhang J. (2020). Disease stage-associated alterations in learning and memory through the electroacupuncture modulation of the cortical microglial M1/M2 polarization in mice with alzheimer’s disease. *Neural Plasticity*.

[26] Yu C. C., Wang J., Ye S. S. (2020). Preventive electroacupuncture ameliorates D-galactose-induced alzheimer’s disease-like pathology and memory deficits probably via inhibition of GSK3*β*/mTOR signaling pathway. *Evidence-based Complementary and Alternative Medicine: eCAM*.

[27] He C., Huang Z. S., Yu C. C. (2021). Preventive electroacupuncture ameliorates D-galactose-induced Alzheimer’s disease-like inflammation and memory deficits, probably via modulating the microbiota-gut-brain axis. *The Iranian Journal of Basic Medical Sciences*.

[28] Wang J., Cheng K., Qin Z. (2017). Effects of electroacupuncture at Guanyuan (CV 4) or Sanyinjiao (SP 6) on hypothalamus-pituitary-ovary axis and spatial learning and memory in female SAMP8 mice. *Traditional Chinese Medicine*.

[29] Jia Y., Zhang X., Yu J. (2017). Acupuncture for patients with mild to moderate Alzheimer’s disease: a randomized controlled trial. *BMC Complementary and Alternative Medicine*.

[30] Yu C. C., He C., Du Y. J. (2021). Preventive electroacupuncture reduces cognitive deficits in a rat model of D-galactose-induced aging. *Neural regeneration research*.

[31] Jiang J., Liu G., Shi S., Li Z. (2016). Musical electroacupuncture may Be a better choice than electroacupuncture in a mouse model of alzheimer’s disease. *Neural Plasticity*.

[32] Tang Y. S., Cao J., Li Z. G. (2014). Effects of music electro-acupuncture and pulsed electro-acupuncture on behavioral changesand the serum *β*-amyloid protein in SAMP8 (senescence accelerated mouse prone 8) mice. *Journal of Alternative & Complementary Medicine*.

[33] Li W., Kong L. H., Wang H. (2016). High-frequency electroacupuncture evidently reinforces hippocampal synaptic transmission in Alzheimer’s disease rats. *Neural Regeneration Research*.

[34] Yu C. C., Wang Y., Shen F. (2018). High-frequency (50 Hz) electroacupuncture ameliorates cognitive impairment in rats with amyloid beta 1-42-induced Alzheimer’s disease. *Neural Regeneration Research*.

[35] Yang Q., Zhu S., Xu J. (2018). Effect of the electro-acupuncture on senile plaques and its formation in APP+/PS1+ double transgenic mice. *Genes & Diseases*.

